# Diagnostic Value of Deep Learning-Based CT Feature for Severe Pulmonary Infection

**DOI:** 10.1155/2021/5359084

**Published:** 2021-11-26

**Authors:** Tinglong Huang, Xuelan Zheng, Lisui He, Zhiliang Chen

**Affiliations:** Department of Critical Care Medicine, The Second Affiliated Hospital of Fujian Medical University, Quanzhou 362000, Fujian, China

## Abstract

The study aimed to explore the diagnostic value of computed tomography (CT) images based on cavity convolution U-Net algorithm for patients with severe pulmonary infection. A new lung CT image segmentation algorithm (U-Net+ deep convolution (DC)) was proposed based on U-Net network and compared with convolutional neural network (CNN) algorithm. Then, it was applied to CT image diagnosis of 100 patients with severe lung infection in The Second Affiliated Hospital of Fujian Medical University hospital and compared with traditional methods, and its sensitivity, specificity, and accuracy were compared. It was found that the single training time and loss of U-Net + DC algorithm were reduced by 59.4% and 9.8%, respectively, compared with CNN algorithm, while Dice increased by 3.6%. The lung contour segmented by the proposed model was smooth, which was the closest to the gold standard. Fungal infection, bacterial infection, viral infection, tuberculosis infection, and mixed infection accounted for 28%, 18%, 7%, 7%, and 40%, respectively. 36%, 38%, 26%, 17%, and 20% of the patients had ground-glass shadow, solid shadow, nodule or mass shadow, reticular or linear shadow, and hollow shadow in CT, respectively. The incidence of various CT characteristics in patients with fungal and bacterial infections was statistically significant (*P* < 0.05). The specificity (94.32%) and accuracy (97.22%) of CT image diagnosis based on U-Net + DC algorithm were significantly higher than traditional diagnostic method (75.74% and 74.23%), and the differences were statistically significant (*P* < 0.05). The network of the algorithm in this study demonstrated excellent image segmentation effect. The CT image based on the U-Net + DC algorithm can be used for the diagnosis of patients with severe pulmonary infection, with high diagnostic value.

## 1. Introduction

At present, the incidence of postoperative pulmonary infection is very high [1]. If the diagnosis is not timely, it is easy to miss the best treatment time. Studies have shown that if the diagnosis can be made in advance, the survival rate of patients with pulmonary infection can be increased by about 40% [2, 3]. Therefore, early and accurate diagnosis of pulmonary infection has become a key issue to improve the cure rate [4, 5]. The main pathogens are bacteria, fungi, viruses, parasites, etc. In addition to pathogen testing, computed tomography (CT) imaging diagnosis has become a common and important method for medical diagnosis. However, as the main feature of judging pulmonary infection, lung CT signs are particularly important from the clarity of lung images and the accurate expression of lung information. Traditional medical image segmentation extracts lung information according to the shallow features of the image and depends on the judgment of the doctor [6]. The addition of subjective factors leads to inaccurate segmentation. Lu et al. [7] proposed a fuzzy logic technology to determine the threshold to achieve accurate segmentation of melanin, but the segmentation effect is poor and inefficient.

With the development of artificial intelligence and information, convolution neural network is introduced into the segmentation of medical images. Nasrullah et al. [8] proposed and used it in the semantic segmentation of natural images and made great progress at that time. In the past segmentation experience, it has exceeded the traditional segmentation method, but its shortcomings cannot be ignored. The excessive multiples adopted in the upsampling operation cause the segmentation accuracy to be not high enough, and the context information is not fully integrated, resulting in low accuracy and precision, which will have a great impact on the survival rate of subsequent diagnosis and posttreatment [9, 10]. The fully convolutional neural network has made great contributions to this problem. As a representative of fully convolutional neural networks, U-Net network can make good use of lower-level information and fuse high-level information when sampling operations [11]. In the following studies, some network structures with better performance are combined with the U-Net network. Baek et al. [12] modified the U-Net to strengthen the position of the feature map, so as to improve the accuracy of extracting the segmentation contour. The 3DU-Net model improves the segmentation performance again by learning the spatial information of the image [13]. In this work, a new lung CT image segmentation algorithm was proposed by adding cavity convolution on the basis of U-Net network. Compared with CNN algorithm, it is applied to the diagnosis of 100 patients with severe pulmonary infection. The sensitivity, specificity, and accuracy of diagnosis are compared with the traditional diagnostic method. It is hoped to provide some theoretical reference for the diagnosis of CT images based on cavity convolution U-Net algorithm in patients with severe pulmonary infection.

## 2. Materials and Methods

### 2.1. Research Objects

In this study, 100 patients with severe pulmonary infection in hospital from July 2019 to July 2021 were enrolled. There were 46 males and 54 females, aged 20–66 years. CT image features based on U-Net + DC algorithm were used to diagnose patients with severe pulmonary infection, which was compared with those of traditional diagnostic methods. The study was approved by the Medical Ethics Committee of Hospital. Patients and their families were informed of the study and signed informed consent.

Inclusion criteria were as follows: (1) separate the same pathogen twice in succession from patient sputum; (2) patients with lung invasive lesions showed by chest X-ray; (3) patients with cough, expectoration, and rales; (4) patients with pathogens isolated from blood or pleural effusion.

Exclusion criteria were as follows: (1) patients who did not sign the informed consent; (2) patients with incomplete clinical data; (3) patients who dropped out of the experiment for personal reasons.

### 2.2. Lung CT Image Segmentation Based on U-Net and Cavity Convolution

The ability of deep learning to extract features is beyond reach of previous machine learning. On account of the fact that the ability of U-Net network to process and integrate high-level and low-level information is better than that of CNN, it is widely used in medical image segmentation. In order to achieve the segmentation of lung CT images, this paper adds cavity deep convolution (DC) on the basis of U-Net network, simplifies and improves the U-Net network, and adds an activation function to increase the nonlinearity of the model. A new lung CT image segmentation algorithm (U-Net + DC) is proposed. The U-Net network is different from the convolution block of the network model proposed in this paper as shown in Figure 1. The convolution block of the network model proposed in this paper is less than the convolution block of the U-Net network by one convolution and an activation function, and the convolution block uses an empty convolution, which can simplify the structure, increase the receptive field, and improve the ability to extract information.

The convolution process of a two-dimensional image can be represented as

(1) $$\begin{array}{c} o\left(a,b\right)=\left(i\times k\right)\left(a,b\right)=\sum_{c}\sum_{d}i\left(c+a,d+b\right)\times k\left(c,d\right). \end{array}$$

In equation (1), *i* is input, *k* is convolution kernel, and *o* is output. When (*a, b*), (*c, d*) is the size of the input image to select the convolution kernel, a smaller convolution kernel is usually selected, which can not only reduce the number of parameters but also increase nonlinearity. The total parameters *p* are as follows:

(2) $$\begin{array}{c} P=\omega +B=k^{2}\times C\times N+N. \end{array}$$

In equation (2), *ω* is the weight, *B* is the partial value, *C* is the number of characteristic channels, and *N* is feature mapping. As a special convolution, cavity convolution can increase the nonlinearity of the model. The essence is to add holes in the convolution and increase the receptive field under the condition of keeping the number of parameters unchanged, which is of great significance to improve the accuracy of image segmentation.  Figure 2 shows the schematic diagram of cavity convolution [14].

Because of the interval of empty convolution, it may cause information discontinuity in practical applications, especially when the image is small and the interval is too large. To solve this problem, this paper designs the cavity size according to Hybrid Dilated Convolution (HDC) standard, which needs to meet the following equation:

(3) $$\begin{array}{c} m_{n}=mix\left[m_{n+1}-2r_{n},m_{n}-2\left(m_{n+1}-r_{n}\right),r_{n}\right]. \end{array}$$

In equation (3), *m*_*n*_ is the largest void spacing before the *n* layer and *r*_*n*_ is the void interval of the *n* layer. The last layer the void spacing selected in this article is (1,2,5).

The pooling layer is downsampling, and the reverse pooling layer is upsampling on the contrary. If it is the maximum pooling *m*_*n*_=*r*_*n*_ in the network transformation process, the location of the activation value is recorded. On the contrary, the location of the nonmaximum is set to 0. Maximum pooling and antipooling are shown in Figure 3.

In this study, the classification output uses *sigmoid* function, which is very sensitive between [−4,4], especially for subtle changes in data that feel very strong. It can be expressed as follows:

(4) $$\begin{array}{c} Sigmoid=\frac{1}{e^{-a}}=\frac{1}{1+e^{-\left(\omega x+c\right)}},\\ Sigmoid^{\prime }\left(a\right)=\frac{e^{-a}}{{\left(1+e^{-a}\right)}^{2}}. \end{array}$$

There are also some problems in the *sidmoid* function. When the number of layers increases, the gradient disappears. The reverse transfer process is as follows:

(5) $$\begin{array}{c} \frac{\partial c}{\partial f_{k}}=Sigmoid^{\prime }\left(a_{k}\right)\omega_{k+1}Sigmoid^{\prime }\left(a_{k+1}\right)\omega_{k+2}\ldots Sigmoid^{\prime }\left(a_{n}\right)\frac{\partial c}{\partial h_{k}}, \end{array}$$

(6) $$\begin{array}{c} h_{k}=Sigmoid\left(a_{n}\right)=Sigmoid\left(\omega_{n}a_{n-1}+f_{n}\right). \end{array}$$

In equation (5), ∂*c*/∂*f*_*k*_ is the gradient of the function to the bias term and *a*_*n*_ is the output.

The Relu function can solve the problem of gradient disappearance, and the convergence rate is fast. The expression is as follows:

(7) $$\begin{array}{c} \text{Relu}\left(x\right)=\max\left(0,x\right),\\ {\text{Relu}}^{\prime }\left(x\right)=\left\{\begin{array}{c} 0,x<0\\ 1,x>0 \end{array}\right.. \end{array}$$

The loss function can increase the robustness of the model, which is crucial to the optimization of the model. The expression of mean square error loss *D* function is shown in the following equation:

(8) $$\begin{array}{c} D=\frac{1}{2n}{\sum \left(y-F\left(i\right)\right)}^{2}. \end{array}$$

In equation (8), *F*(*i*) is the output of the model. Then, activation function is as follows:

(9) $$\begin{array}{c} Sigmoid\left(Z\right)=Sigmoid\left(\omega A+b\right). \end{array}$$

In equation (9), *A* and *Z* are the input and output of the last layer and *b* is the offset. However, compared with the mean square error loss function, the cross entropy loss function and the Sigmoid function are better. So this paper selects the cross entropy loss function, and its expression is shown in the following equation:

(10) $$\begin{array}{c} D=\frac{1}{n}\sum \left[y\;\log\left(F\left(i\right)\right)+\left(1-y\right)\log\left(1-F\left(i\right)\right)\right]. \end{array}$$

Image denoising and data enhancement are needed before training. Curvature-driven denoising method is used in this paper. Curvature-driven minimization energy function is as follows:

(11) $$\begin{array}{c} G\left(v\right)=\lambda \int_{\Omega }\left|h_{v}\right|\text{d}x+\int_{\Omega }{\left(F-v\right)}^{2}\text{d}x. \end{array}$$

In equation (11), (*x*, *y*, *v*(*x*, *y*)) is a surface, (*x*, *y*, *F*(*x*, *y*)) is the input image, and *λ* is the parameter. The regularization *h*_*v*_ is expressed as follows:

(12) $$\begin{array}{c} h_{v}=\frac{1}{2}\nabla \left(\frac{\nabla v}{\sqrt{1+{\left|\nabla v\right|}^{2}}}\right). \end{array}$$

According to the corresponding Euler-Lagrange function, curvature smoothing is realized. In order to improve the convergence speed, we choose Z-score standardized processing:

(13) $$\begin{array}{c} x_{1}=\frac{x_{2}-\bar{x}}{\sigma }. \end{array}$$

In equation (13), $\bar{x}$ is the mean and *σ* is the standard deviation. The data enhancement increases the robustness and generalization ability of the model to prevent the occurrence of overfitting. The enhancement methods selected in this paper are rotation, flip, offset, scaling, elastic transformation, and so on. The original data is extended to about 20,000, and it is trained. The image segmentation process constructed in this paper is shown in Figure 4.

### 2.3. Simulation Experiment

Simulation environment: the operating system is Windows 10 on LINUX, the processor is Xeon CPU E5-2630, the display card is NVIDIA Quadro K2200, the framework is TensorFlow and Keras, the language is Python 3.5, and the visual library is OpenCV, SimpleITK, CUDA9.0, cudnn, etc.

Network parameters: input image resolution is 256256, convolution block is a hole convolution and activation function, convolution kernel size is 33, according to HDC principle, hole interval is (1,2,5), activation function is Relu function, with 2 × 2 maximum pooling downsampling, 1 × 1 convolution layer for multichannel feature fusion, 3 × 3 convolution upsampling, and the number of training in this paper is 60.

In this study, the lung CT image data is used as the simulation object, and the CNN algorithm is introduced to compare with the algorithm in this paper. The measurement index is Dice coefficient [15].

(14) $$\begin{array}{c} \text{Dice}=\frac{2\left|E\cap F\right|}{\left|E\right|+\left|F\right|}. \end{array}$$

In equation (14), *E* is the gold standard for the segmentation of pulmonary nodules, *F* is the segmentation result, and the range of Dice coefficient is [0,1]. The larger the value is, the better the algorithm performance is.

### 2.4. CT Examination and Radiofrequency Ablation

At the beginning of scanning, the patient was supine in the center of the CT examination bed. The patient should maintain a peaceful state of mind, not move the body, and routinely inhale. Scanning ranges from chest entrance to diaphragm. Scanning parameters: CT tube voltage is 120 kV, tube current is 300 mAs, scanning field is 260∼360 mm, matrix is 512512, layer thickness is 4 mm, and layer spacing is 4 mm. Siemens CT tube voltage is 120 kV, tube current is 380 mAs, scanning field is 220∼280 mm, matrix is 512512, layer thickness is 2 mm, and layer spacing is 2 mm. All patients underwent plain scan. CT image is uploaded to Siemens for readings, window width of lung window is 1 600, window level of lung window is 400, and window width of Mediastinal window is 350. The CT images were reviewed by two experienced physicians respectively, and conclusions were reached through discussion in case of disagreement.

### 2.5. Observation Indicators

The types of pathogens, morphological characteristics of CT manifestations, and lesion distribution of patients with severe pulmonary infection were recorded, and the incidence of morphological characteristics of CT manifestations of pulmonary infection with different pathogens was compared. The sensitivity, specificity, and accuracy of traditional method diagnosis and CT image diagnosis based on U-Net + DC algorithm were compared and calculated.

(15) $$\begin{array}{c} \text{sensitivity}=\frac{\text{TP}}{\text{TP}+\text{FN}}\times 100\%, \end{array}$$

(16) $$\begin{array}{c} \text{specificity}=\frac{\text{TN}}{\text{TN}+\text{FN}}\times 100\%, \end{array}$$

(17) $$\begin{array}{c} \text{accuracy rate}=\frac{\text{TP}+\text{TN}}{\text{Total}}\times 100\%. \end{array}$$

In equations (15), (16), and (17), TP represents true positive, TN represents true negative, FP represents false positive, and FN represents false negative.

### 2.6. Statistical Methods

The data in this study were analyzed by SPSS 22.0 statistical software. The measurement data were expressed as mean ± standard deviation ($\bar{x}\pm s$), and the count data were expressed as percentage (%). The difference was statistically significant with *P* < 0.05.

## 3. Results

### 3.1. Algorithm Simulation Effects

Figure 5 shows the changes in the Loss value and Dice of the U-Net + DC model as the number of iterations increased. It was noted that when the number of iterations was 30, the Loss value tended to be stable, and finally, the Loss value reached 0.0659, and Dice increased with the number of iterations and, finally, reached 0.9495.

Figure 6 shows the single training time of the two algorithms. It was noted that the single training time of the CNN algorithm was 690 s, and the single training time of the U-Net + DC algorithm was 280 s. The single training time of the U-Net + DC algorithm was significantly less than the single training time of the CNN algorithm by 59.4%, and the difference was statistically significant (*P* < 0.05).

Figure 7 shows the Loss value and Dice coefficient of the two algorithms. It was noted that the Loss value and Dice of the CNN algorithm were 0.0731 and 0.9387, respectively, and the Loss value and Dice of the U-Net + DC algorithm were 0.0659 and 0.9495, respectively. The Loss value of the U-Net + DC algorithm was smaller than the Loss value of the CNN algorithm by 9.8%, and the difference was statistically significant (*P* < 0.05). The Dice of the U-Net + DC algorithm was larger than the Dice of the CNN algorithm by 3.6%, and the difference was statistically significant (*P* < 0.05). It showed that, with the gold standard as a reference, the Loss value and Dice of the U-Net + DC algorithm were improved versus the CNN algorithm, and its segmentation effect was better than that of the CNN algorithm.

### 3.2. Comparison of Lung CT Image Segmentation Effects of the Two Algorithms

Figure 8 shows the lung CT image segmentation effects of the two algorithms. It was noted that, with the gold standard as a reference, the edges segmented by the CNN algorithm were blurred, and the segmentation was affected by the fine blood vessels of the lung organs and other tissue, while the outline of the lungs segmented by the U-Net + DC algorithm was more accurate, and the edges were smoother, which was closer to the gold standard.

### 3.3. Types and Morphological Characteristics of Pathogens in Patients with Severe Lung Infections

Figure 9 shows the pathogens in patients with severe lung infections. Of the 100 patients with severe lung infections, 28% (28 cases) had fungal infections, 18% (18 cases) had bacterial infections, 7% (7 cases) had viral infections, 7% (7 cases) had tuberculosis infections, and 40% (40 cases) had mixed infections, accounting for the highest proportion.

Figure 10 shows the CT morphological characteristics of severe lung infections. Of the 100 patients with severe pulmonary infections, 36% (36 cases) had ground-glass shadows, 38% (38 cases) had consolidation shadows, 26% (26 cases) had nodules or masses, 17% (17 cases) had reticulated or linear shadows, and 20% (20 cases) had hollow shadows.

### 3.4. Images of Various Morphological Features of Patients with Severe Lung Infections

Figure 11 shows images of various morphological features of patients with severe lung infections.  Figure 11(a) shows the ground-glass shadow of the right lung.  Figure 11(b) shows the large consolidation shadows of the lungs.  Figure 11(c) shows the mass-like high-density shadows of the upper lobe of the left lung, and the lungs had multiple small nodules with clear boundaries.  Figure 11(d) shows ground-glass shadows and fine mesh shadows.  Figure 11(e) shows a hollow shadow in the upper right lung, with patches of increased density around it.

### 3.5. The Distribution of Lesions in Patients with Severe Lung Infections

Figure 12 shows the lesion distribution of patients with severe lung infections. It was noted that there were 20 cases, 10 cases, 3 cases, and 3 cases with subpleural distribution, middle internal zone distribution, diffuse distribution, and irregular distribution in patients with ground-glass shadows in CT; of the patients with consolidation shadows in CT, there were 21, 8, 5, and 4 cases with subpleural distribution, midinternal zone distribution, diffuse distribution, and irregular distribution, respectively; of the patients with nodules or masses in CT, there were 10 cases, 3 cases, 12 cases, and 1 case with the subpleural distribution, the middle and inner zone distribution, the diffuse distribution, and the irregular distribution, respectively; of the patients with network or line-like shadows in CT, there were 12 cases, 1 case, 3 cases, and 2 cases with the subpleural distribution, the middle inner zone distribution, the diffuse distribution, and irregular distribution, respectively; of the patients with hollow shadows in CT, there were 13 cases, 1 case, 4 cases, and 3 cases with subpleural distribution, midinternal zone distribution, diffuse distribution, and irregular distribution, respectively.

### 3.6. Comparison of the Incidence of Different CT Morphological Characteristics of Lung Infections with Different Pathogens

Figure 13 shows the incidence of different CT morphological characteristics lung infections with different pathogens. It was noted that the incidence of ground-glass shadows, consolidation shadows, nodules or mass shadows, network or line-like shadows, and hollow shadows in patients with fungal infections was 25%, 25%, 14.3%, 7.1%, and 28.6, respectively; the incidence of ground-glass shadow, consolidation shadow, nodule or mass shadow, network or linear shadow, and hollow shadow in patients with bacterial infections was 16.7%, 5.6%, 44.4%, 22.2%, and 11.1%, respectively. There were statistically significant differences in the incidence of ground-glass shadows, consolidation shadows, nodules or mass shadows, network or line-like shadows, and hollow shadows in patients with fungal and bacterial infections (*P* < 0.05).

### 3.7. Diagnosis Accuracy of Patients with Severe Lung Infection in Two Ways

Figure 14 shows the sensitivity, specificity, and accuracy of the two methods of diagnosis. It was noted that the sensitivity of the traditional method was 88.31%, the specificity was 75.74%, and the accuracy was 74.23%; the sensitivity of CT image diagnosis based on the U-Net + DC algorithm was 98.13%, the specificity was 94.32%, and the accuracy was 97.22%; the specificity and accuracy of CT image diagnosis based on U-Net + DC algorithm were significantly higher than those of traditional method, and the difference was *statistically* significant (*P* < 0.05).

## 4. Discussion

At present, the morbidity and mortality of patients after the surgery are extremely high due to severe lung infections [16]. CT imaging plays an important role in the diagnosis of severe pulmonary infections and there are high requirements on the accuracy and resolution of the images. With the rapid development of artificial intelligence and information technology, the application of deep learning in medical imaging has made great contributions to the segmentation and diagnosis of medical images [17, 18]. In this study, DC was incorporated into the U-Net network to simplify and improve the U-Net network, and then the improved one was used to process the lung CT images, and its segmentation effect was compared with that of the CNN algorithm. The results showed that the U-Net + DC algorithm had shorter single training time and a lower Loss value than the CNN algorithm, and the difference was statistically significant (*P* < 0.05). Specifically, the single training time was reduced by 59.4% and the Loss value was reduced by 9.8%. The Dice of the U-Net + DC algorithm was larger than the Dice of the CNN algorithm by 3.6%, and the difference was statistically significant (*P* < 0.05). It showed that, with the gold standard as a reference, the U-Net + DC algorithm's various indicators were improved versus the CNN algorithm. It can segment the contours of the lungs more accurately, and the edges were smoother, which was closer to the gold standard.

After that, it was applied to the diagnosis of 100 patients with severe lung infections, and it was compared with the traditional method for the sensitivity, specificity, and accuracy of the diagnosis. The results found that, of the 100 patients with severe lung infections, 28% (28 cases) had fungal infections, 18% (18 cases) had bacterial infections, 7% (7 cases) had viral infections, 7% (7 cases) had tuberculosis infections, and 40% (40 cases) had mixed infections, accounting for the highest proportion. This was in line with the results of Suleyman et al. [19] that, of the 88 patients with lung infections after hematopoietic stem cell transplantation, 27 cases had fungal infections, 12 cases had bacterial infections, and 88 cases had viral infections. Of the 36 patients with ground-glass shadows in CT, there were 20 cases, 10 cases, 3 cases, and 3 cases with subpleural distribution, middle internal zone distribution, diffuse distribution, and irregular distribution; of the 38 patients with consolidation shadows in CT, there were 21, 8, 5, and 4 cases with subpleural distribution, midinternal zone distribution, diffuse distribution, and irregular distribution, respectively; of the 26 patients with nodules or masses in CT, there were 10 cases, 3 cases, 12 cases, and 1 case with the subpleural distribution, the middle and inner zone distribution, the diffuse distribution, and the irregular distribution, respectively; of the 17 patients with network or line-like shadows in CT, there were 12 cases, 1 case, 3 cases, and 2 cases with the subpleural distribution, the middle inner zone distribution, the diffuse distribution, and irregular distribution, respectively; of the 20 patients with hollow shadows in CT, there were 13 cases, 1 case, 4 cases, and 3 cases with subpleural distribution, midinternal zone distribution, diffuse distribution, and irregular distribution, respectively. This was consistent with the results of Ioannou et al. [20] that 4 out of 10 cases of *Aspergillus* infection had subpleural wedge-shaped consolidation shadows. The incidence of ground-glass shadows, consolidation shadows, nodules or mass shadows, network or line-like shadows, and hollow shadows in patients with fungal infections was 25%, 25%, 14.3%, 7.1%, and 28.6, respectively; the incidence of ground-glass shadow, consolidation shadow, nodule or mass shadow, network or linear shadow, and hollow shadow in patients with bacterial infections was 16.7%, 5.6%, 44.4%, 22.2%, and 11.1%, respectively. There were statistically significant differences in the incidence of ground-glass shadows, consolidation shadows, nodules or mass shadows, network or line-like shadows, and hollow shadows in patients with fungal and bacterial infections (*P* < 0.05). The specificity (94.32%) and accuracy (97.22%) of CT image diagnosis based on U-Net + DC algorithm were significantly higher than those of traditional method (75.74% and 74.23%), and the differences were statistically significant (*P* < 0.05). This is better than Chung et al. [21]. The addition of deep learning algorithm makes the diagnosis and segmentation of severe lung patients more accurate and helps medical staff to control the disease more effectively, so as to better treat it.

## 5. Conclusion

In this study, the DC was incorporated into the U-Net network to simplify and improve the U-Net network, and the improved algorithm was used to process lung CT images, and then it was compared with the CNN algorithm for the sensitivity, specificity, and accuracy of diagnosis. The results showed that the network of the algorithm in this study had better image segmentation effects; in medical diagnosis, CT images based on U-Net + DC algorithm can be used to diagnose severely infected patients, demonstrating high diagnostic value. However, some limitations in the study should be noted. The sample size is small, which will reduce the power of the study. In the followup, expanded sample size is necessary to strengthen the findings of the study. In conclusion, CT images based on hollow convolution U-Net algorithm are analyzed, which improves the segmentation effect of images and provides a new direction for the diagnosis of patients with severe pulmonary infection.

## Figures and Tables

**Figure 1:** Comparison of two network convolution blocks. (a) U-Net network convolution blocks. (b) U-Net + DC model convolution block proposed in this paper.

**Figure 2:** Schematic of cavity convolution.

**Figure 3:** Maximum pooling and reverse pooling.

**Figure 4:** Construction of algorithm segmentation flow.

**Figure 5:** Changes in Loss value and Dice coefficient of U-Net + DC model under different iterations.

**Figure 6:** Comparison of single training time of the two algorithms. *Note.*^*∗*^ indicates that the difference was statistically significant compared to the CNN algorithm (*P* < 0.05).

**Figure 7:** Comparison of Loss value and Dice of the two algorithms. *Note.*^*∗*^ indicates that the difference was statistically significant compared to the CNN algorithm (*P* < 0.05).

**Figure 8:** Comparison of lung CT image segmentation results of the two algorithms. (a) The original image, (b) the gold standard, (c) the CNN segmentation result, and (d) the U-Net + DC segmentation result.

**Figure 9:** The types of pathogens in patients with severe lung infections.

**Figure 10:** CT morphological characteristics of patients with severe lung infections.

**Figure 11:** Various morphological feature images of patients with severe lung infections. (a) Ground-glass shadow, (b) consolidation shadow, (c) nodule or mass shadow, (d) network or line-like shadow, and (e) hollow shadow.

**Figure 12:** The distribution of lesions in patients with severe lung infections.

**Figure 13:** Comparison of the incidence of different CT morphological characteristics of lung infections with different pathogens. *Note.*^*∗*^ means the difference was statistically significant compared to fungal infections (*P* < 0.05).

**Figure 14:** Comparison of the sensitivity, specificity, and accuracy of the two diagnosis methods. (a) Traditional method diagnosis. (b) CT image diagnosis based on U-Net + DC algorithm. *Note.*^*∗*^ indicates that, compared with the traditional method, the difference was statistically significant (*P* < 0.05).

## Data Availability

The data used to support the findings of this study are available from the corresponding author upon request.

## References

[1] Shen J., Huang L., Hao C. (2020 Oct). Value of multi‐slice spiral computed tomography for diagnosis of tracheobronchial foreign body aspiration in children: 5‐year retrospective study. *Pediatrics International*.

[2] Huang C., Huang L., Wang Y. (2021 Jan 16). 6-month consequences of COVID-19 in patients discharged from hospital: a cohort study. *The Lancet*.

[3] Jin L., Chang K. (2021 Jul 7). Optimized fuzzy C-means algorithm-based coronal magnetic resonance imaging scanning in tracheal foreign bodies of children. *J Healthc Eng*.

[4] Fernández-de-las-Peñas C., Gómez-Mayordomo V., García-Azorín D. (2021 Jun 28). Previous history of migraine is associated with fatigue, but not headache, as long-term post-COVID symptom after severe acute respiratory SARS-CoV-2 infection: a case-control study. *Frontiers in Human Neuroscience*.

[5] Xu X., Yu C., Qu J. (2020 May). Imaging and clinical features of patients with 2019 novel coronavirus SARS-CoV-2. *European Journal of Nuclear Medicine and Molecular Imaging*.

[6] Shaw B., Daskareh M., Gholamrezanezhad A. (2021 Jan). The lingering manifestations of COVID-19 during and after convalescence: update on long-term pulmonary consequences of coronavirus disease 2019 (COVID-19). *La radiologia medica*.

[7] Lu M. T., Raghu V. K., Mayrhofer T., Aerts H. J. W. L., Hoffmann U. (2020 Nov 3). Deep learning using chest radiographs to identify high-risk smokers for lung cancer screening computed tomography: development and validation of a prediction model. *Annals of Internal Medicine*.

[8] Nasrullah N., Sang J., Alam M. S., Mateen M., Cai B., Hu H. (2019 Aug 28). Automated lung nodule detection and classification using deep learning combined with multiple strategies. *Sensors*.

[9] Kottlors J., Geissen S., Jendreizik H. (2021 Jun 1). Contrast-enhanced black blood MRI sequence is superior to conventional T1 sequence in automated detection of brain metastases by convolutional neural networks. *Diagnostics*.

[10] Lee S.-A., Jo S.-W., Chang S.-K., Kwon K.-H. (2021 Apr 24). Improvement of the diagnostic performance of facial neuritis using contrast-enhanced 3D T1 black-blood imaging: comparison with contrast-enhanced 3D T1-spoiled gradient-echo imaging. *Journal of Clinical Medicine*.

[11] Wan Z., Dong Y., Yu Z., Lv H., Lv Z. (2021 Jul 9). Semi-supervised support vector machine for digital twins based brain image fusion. *Frontiers in Neuroscience*.

[12] Baek S., He Y., Allen B. G. (2019 Nov 21). Deep segmentation networks predict survival of non-small cell lung cancer. *Scientific Reports*.

[13] Lv Z., Qiao L., Wang Q., Piccialli F. (2020 Jul 17). Advanced machine-learning methods for brain-computer interfacing. *IEEE/ACM Transactions on Computational Biology and Bioinformatics*.

[14] Mattonen S. A., Davidzon G. A., Bakr S. (2019 Mar). [18F] FDG positron emission tomography (PET) tumor and penumbra imaging features predict recurrence in non-small cell lung cancer. *Tomography*.

[15] Hu M., Zhong Y., Xie S., Lv H., Lv Z. (2021 Jul 30). Fuzzy system based medical image processing for brain disease prediction. *Frontiers in Neuroscience*.

[16] Chen Y., Bai J. (2020 Sep). Maternal and infant outcomes of full-term pregnancy combined with COVID-2019 in Wuhan, China: retrospective case series. *Archives of Gynecology and Obstetrics*.

[17] Ather S., Kadir T., Gleeson F. (2020 Jan). Artificial intelligence and radiomics in pulmonary nodule management: current status and future applications. *Clinical Radiology*.

[18] Chrzan R., Bociąga-Jasik M., Bryll A., Grochowska A., Popiela T. (2021 May 10). Differences among COVID-19, bronchopneumonia and atypical pneumonia in chest high resolution computed tomography assessed by artificial intelligence technology. *Journal of Personalized Medicine*.

[19] Suleyman G., Fadel R. A., Malette K. M. (2020 Jun 1). Clinical characteristics and morbidity associated with coronavirus disease 2019 in a series of patients in metropolitan detroit. *JAMA Network Open*.

[20] Ioannou G. N., Locke E., Green P. (2020 Sep 1). Risk factors for hospitalization, mechanical ventilation, or death among 10 131 US veterans with SARS-CoV-2 infection. *JAMA Network Open*.

[21] Chung M., Bernheim A., Mei X. (2020 Apr). CT imaging features of 2019 novel coronavirus (2019-nCoV). *Radiology*.

